# Research on Ultrasonic Image Recognition Based on Optimization Immune Algorithm

**DOI:** 10.1155/2021/5868949

**Published:** 2021-05-17

**Authors:** Xueqiang Zeng, Sufen Chen

**Affiliations:** ^1^School of Computer & Information Engineering, Jiangxi Normal University, Nanchang 330022, China; ^2^School of Information Engineering, Nanchang Institute of Technology, Nanchang 330099, China

## Abstract

With the rapid development of science and technology, ultrasound has been paid more and more attention by people, and it is widely used in engineering, diagnosis, and detection. In this paper, an ultrasonic image recognition method based on immune algorithm is proposed for ultrasonic images, and its method is applied to medical ultrasound liver image recognition. Firstly, this paper grays out the ultrasound liver image and selects the region of interest of the image. Secondly, it extracts the feature based on spatial gray matrix independent matrix, spatial frequency decomposition, and fractal features. Then, the immune algorithm is used to classify and identify the normal liver, liver cirrhosis, and liver cancer ultrasound images. Finally, based on the deficiency of the immune algorithm, it is combined with the support vector machine to form an optimized immune algorithm, which improves the performance of ultrasonic liver image classification and recognition. The simulation shows that this paper can effectively classify the normal liver, liver cirrhosis, and liver cancer ultrasound images. Compared with the traditional immune algorithm, this paper combines the immune algorithm with the support vector machine, and the optimized immune algorithm can effectively improve the performance of ultrasonic liver image classification and recognition.

## 1. Introduction

Liver diseases threaten human health at all times. The diagnosis and treatment of liver diseases have always been the focus of medical research. At present, diseases caused by liver diseases have become one of the main causes of human death, including liver cancer, fatty liver, and schistosomiasis. If these diseases can be detected at the same time and treated at the same time, the possibility of a cure can be greatly increased.

One of the methods of examining liver disease is the scanning of medical images. B-ultrasound is one of them, it is one of the most widely used and simple clinical applications, and it has been paid more and more attention. Because the B-ultrasound inspection equipment is relatively cheap, the treatment cost is low, there is no adverse reaction, it can be repeatedly checked, and the penetration rate in China is high. B-ultrasound is to display the echo signal as a two-dimensional image in the form of a light spot. The size of the echo is represented by the brightness of the light spot. According to the gray level of the light spot, the two-dimensional structure image with a well-defined layer is a grayscale modulation type. B-ultrasound can obtain various cut-off patterns of various organs in the human body and is more suitable for diagnosis of various organ diseases such as liver, gallbladder, kidney, bladder, uterus, and ovary. Since the ambiguity of B-mode images brings certain difficulties to image recognition, improving the correct recognition rate has been a research hot spot at home and abroad. How to effectively extract information from B-mode images and achieve accurate recognition is the key to improving the diagnostic level.

Therefore, many researchers in China have painstakingly studied how to improve the recognition efficiency and accuracy of ultrasound images and reduce the number of repeated treatments and examinations. This topic needs to be solved urgently, and it also has far-reaching significance.

For a long time, in the process of B-ultrasound image recognition, doctors have established diagnostic experience to analyze and judge pathology through a large number of visual observations, which makes the judgment of images have no objective evaluation criteria, so there is a poor repeatability, and the accuracy is different due to the doctor's diagnosis level. In order to better improve the accuracy and reliability of B-mode image recognition, it is urgent to develop the image recognition function of the ultrasonic diagnostic system. This requires a certain processing of the B-mode image in order to obtain certain quantitative parameters, reducing the errors and workloads that occur when doctors use the naked eye to interpret medical images.

At present, the classification and recognition of liver ultrasound images are the focus and difficulty of many scholars at home and abroad. There are many literatures about the classification of prostate and breast images in the classification of ultrasound images; in particular, for the recognition of breast tumors, many scholars have done a lot of research. This provides a good contrast and reference for our work in the field of liver ultrasound image recognition. The recognition and classification of hyperhepatic images that we have studied is a very challenging subject. In this respect, domestic and foreign scholars have also done some exploratory work. Because of its complexity, ultrasound images have many difficulties in classification. Firstly, the image is noisy and the contrast of the lesion is low, which undoubtedly has a great impact on the effect of feature extraction. Secondly, feature selection is also a huge difficulty, and how to find the case to be identified with a high recognition rate of features is also a problem for many researchers.

In this paper, based on immune algorithm, an ultrasonic image recognition method based on immune algorithm is proposed, which is applied to ultrasonic liver image recognition. An optimized immune algorithm is formed by combining immune algorithm with support vector machine. The main contributions of this paper are as follows.

1. The ultrasonic image of the liver is grayscale, and the region of interest is selected
2. Feature extraction is achieved by spatial gray independent matrix, spatial frequency decomposition, and classification features
3. The ultrasonic images of normal liver, liver cirrhosis, and liver cancer were classified and recognized by immune algorithm, and a method of ultrasonic liver image recognition based on immune algorithm was proposed
4. An optimized immune algorithm is formed by combining immune algorithm with support vector machine

## 2. Related Work

With the development of information technology, researchers combine digital image processing technology, information technology, and medical diagnosis knowledge. Firstly, the digital image processing technology is used to process the medical image, and then, the doctor's knowledge of pathological diagnosis is used to make scientific judgment, which can improve the accuracy and reliability of diagnosis [1–3].

The classification of medical images is to find the law of sample distribution from known training samples and to apply this rule to the identification of new samples. A good classifier can not only better explain the known samples but also make better predictions and judgments on new samples and even unobservable phenomena. This is what is commonly referred to as generalization ability.

At present, more and more researchers use optimization algorithms for medical image recognition. Commonly used algorithms are Particle Swarm Optimization (PSO) [4] and Ant Colony Optimization (ACO) [5], artificial bee colony (ABC) algorithm [6], genetic algorithm [7], simulated annealing algorithm, and immune algorithm. The immune algorithm was inspired by the biological immune mechanism. The earliest immunology dates back more than 200 years. In 1974, Jarne's immune network theory was awarded Nobel, and people began to become interested in immune network theory. Edward Jenner discovered the vaccinia vaccine in 1796 and used it to treat the deadly infectious disease of human smallpox. In 1986, Farmer's paper “Immune System, Adaptation and Machine Learning” first developed the immune mechanism and artificial intelligence, and then, the artificial immune system was officially put on the road. In the early 1990s, Bersini added AI ideas to the control problem [8]. In 1990, Ishida introduced AI in the problem of fault diagnosis [9]. After 1999, Castro and Gaspar designed two algorithms based on the principle of clonal selection: clonal selection algorithm and pattern tracking algorithm [10]. In the same year, Dasgupta and other scholars designed a negative selection algorithm using the negative selection mechanism of immune tolerance alone [11]. These algorithms are based on the initial biological immune mechanisms that have emerged in just a few decades, and it can be seen that immunology has great potential to solve problems. More research and application of immunology theory is the development trend of today's high-end field.

An immune algorithm is an algorithm that is based on the principles of immunology and is used in engineering applications. The development of immunology has been continuously advanced through the successive submission of various immune algorithms. Because the immune algorithm is a problem-oriented method, the new algorithm is generated based on the relevant principles of the immune system, or the original technology is improved to make it more suitable for engineering applications. Representative examples include Castro's proposed clonal selection algorithm [12] and artificial immune network algorithm [13] and Forrest's negative selection algorithm [14].

The characteristics of the immune algorithm are as follows: each element has intelligence, has high autonomy, and can judge whether other elements are autologous types; the immune system elements selectively recognize nonself types; and diversity is generated by gene combination. Self-learning is at the network component stage, as long as the new nonself appears, nonself learning [15–17]. Identification is a passive approach, trying to identify nonself, and communication between units is the affinity between them, not hard links. The immune algorithm simulates the adaptive and artificial immunity of the human immune system, which is a means to strengthen the human immune system. A concentration-based selection update strategy is adopted to prevent the occurrence of premature phenomenon and ensure that the search process is proceeding toward global optimization. The search target of the immune algorithm has a certain degree of dispersion and independence, and the diversity search is realized.

## 3. Proposed Method

### 3.1. Ultrasonic Liver Image Preprocessing

In the process of liver hyperimage recognition, feature extraction is the premise of image recognition. In a broad sense, image feature extraction is a kind of transformation, that is, the low-dimensional space is used to represent the high-dimensional image sample space. Feature selection and extraction are very important, which directly affect the design, performance, and accuracy of image recognition classifier. Its basic task is to find out the most effective features from many features. In this chapter, according to the characteristics of liver ultrasound image, the liver ultrasound image is preprocessed, including transforming the image into gray image and extracting the region of interest (ROI) [18].

#### 3.1.1. Characteristics of Ultrasound Liver Images

First, the ultrasonographic features of normal liver, liver cirrhosis, and liver cancer are described as follows.

1. Ultrasound images of normal liver showed fine light spots and uniform distribution of liver parenchyma, sometimes sparse, scattered slightly strong light spots and short linear echoes, and the outline was complete, the boundary was neat, and the boundary was clear. The corresponding image features were described as normal liver texture rules, clear, uniform gray distribution, and its texture distribution was dense
2. Ultrasound medical images of cirrhosis showed uneven, thin wave, stepped and serrated echoes, and the echo light spots in liver parenchyma were coarser and unevenly distributed
3. Ultrasound imaging of liver cancer and low echo sonography of liver parenchyma. The corresponding image features are irregular but fresh, and the range of grayscale distribution increases

In this paper, the description of these features is regarded as the expert experience, combining with the feature descriptors of the region, the feature of never changing moment, the feature of frequency spectrum, the statistical moment feature of texture, and the description of texture based on gray level cooccurrence matrix. The changes of these four kinds of liver tissues were quantified, and the B-ultrasound images were further classified and recognized by these quantized values.

#### 3.1.2. Grayscale Processing

Because of insufficient exposure, the gray change range of the whole image is usually very small. If the gray change of the real scene is really small, in order to increase the contrast of all or part of the image, the gray change range can be enlarged by gray transformation. In this way, the original image with small gradient becomes rich in gray level, which improves the visual perception conditions and achieves the purpose of image enhancement.

#### 3.1.3. Selection of Regions of Interest

Because the current conditions cannot automatically extract the region of interest, the region of interest extraction in this paper is manually extracted under the guidance of doctors with rich clinical experience. Region of interest extraction follows the following principles [19–21].

1. Each image selected two rectangular areas, one located inside the space occupying lesion as A1 and one located in the normal liver as A2
2. A1 and A2 are as far as possible to maintain the same depth, for the fan array probe images, as far as possible in the same arc; for the linear array probe images, as far as possible in the same horizontal position. And A2 is closer to A1 as far as possible
3. A1 and A2 may vary in size. A1 may include as many space-occupying lesions as possible, but not beyond the scope of space-occupying lesions. A2 may be as large as possible within the allowable scope
4. When choosing A2, try to avoid large intrahepatic ducts, such as blood vessels, bile ducts, and gallbladder

### 3.2. Ultrasonic Liver Image Feature Extraction

The entropy, Fourier energy spectrum, angle second-order matrix, and contrast are calculated from the spatial grayscale independent matrix of 1 × 1 cm^2^ region. The *M* band wavelet transform is used to calculate the fractal feature vectors.

The following is the parameter definition: *f*(*i*, *j*) is the density of pixels in ROI.

1. Entropy *H*

(1) $$\begin{array}{c} H=\overset{i-1}{\underset{1}{\sum }}\overset{j-1}{\underset{1}{\sum }}P\left(i,j\right)\log P\left(i,j\right). \end{array}$$

Entropy represents the degree of nonuniformity or complexity of texture in images. When the complexity is high, the entropy value is large; otherwise, the entropy value is smaller or 0 [22].

(2) Angular Second Moment (ASM)

Use spatial grayscale independent matrix (cooccurrence matrix). *C*(*a*, *b*; *d*, *θ*) is a conditional probability function based on second-order estimation, which represents the probability of grayscale from *a* to *b*, *d* is the sampling of the system, and the direction is specified by angle *θ*. The ASM, calculated by *C*(*a*, *b*; *d*, 0°), is defined as follows:

(2) $$\begin{array}{c} C\left(a,b;1,0^{0}\right)=\frac{1}{T\left(1,0^{0}\right)}\text{cardinality}\left\{\left[\left(k,l\right),\left(m,n\right)\right]\in \text{ROI}:\left|k-m\right|=1,l=n,f\left(k,l\right)=a,f\left(m,n\right)=b\right\}. \end{array}$$

*T*(1, 0°) is the total number of pairs of pixels in the ROI, ROI is the sampling interval *d* = 1, and the direction angle is 0°. Get ASM:

(3) $$\begin{array}{c} \text{ASM}=\underset{a}{\sum }\underset{b}{\sum }C\left(a,b;1,0^{\circ }\right). \end{array}$$

Second-order moment is a measure of the uniformity of image gray distribution. When the elements of gray level cooccurrence matrix concentrate on the principal diagonal line, the gray distribution of the image is more uniform from the local area; the whole texture is coarse, and the variance is larger, so the second-order moment is larger. When the texture of the image is more fine and the gray distribution is uniform, the energy value is larger. On the contrary, when the gray distribution of the image is very uneven and rough, the energy value is smaller [23].

(3) Fractal feature vector based on wavelet transform of *M* band

Pyramid-based wavelet transform provides more important features than ordinary multiresolution analysis. Therefore, the fractal feature vectors are based on ordinary multiresolution analysis and are defined as follows:

(4) $$\begin{array}{c} MF\equiv \left(D_{f}^{m,i},D_{f}^{m,i+1},\cdots ,D_{f}^{m-n+1,i},\cdots ,D_{f}^{m-n+1,i+k}\right), \end{array}$$

where *D*_*f*_ is the fractal of the *i*th subimage at level *m*.

For *M* band wavelet transform, *M* takes different values at different levels. The common multiresolution in formula (4) is implemented by a dual channel and 3-channel filter layer hybrid structure. The fractal dimension of the LH band (low-pass filter along abscissa and high-pass filter along ordinate) provides information for cirrhosis and hepatocellular carcinoma, and the characteristic order is as follows:

(5) $$\begin{array}{c} MF\equiv \left(D_{f}^{3,0},D_{f}^{2,1},D_{f}^{2,2},D_{f}^{1,1},D_{f}^{1,2},D_{f}^{1,3},D_{f}^{1,4},D_{f}^{1,5},D_{f}^{1,6}\right), \end{array}$$

where *D*_*f*_^3,0^ is the initial image fractal dimension, *D*_*f*_^2,1^ is the fractal dimension of the LL image, and *D*_*f*_^2,2^ is the fractal dimension of the LH image. The last 6 parts of the eigenvector are calculated from the overdraft diagram.

### 3.3. Immune Algorithm and Support Vector Machine

#### 3.3.1. Working Principle of Immune Algorithm

In mathematical theory, immune algorithm is often used to deal with optimization problems (NBP) [24].  Figure 1 gives the basic work flow of the immune algorithm. The steps in the diagram, such as antigen recognition and parameter determination, coding and initializing antibody groups, and memory cell evolution and recruiting new members, correspond to specific evolutionary processes in the biological immune system. In immunology, these processes are humoral immune responses, and in algorithm, a systematic immune algorithm is formed, that is, the optimization problem is the antigen in immunology. The undetermined solution of NBP is considered as the antibody in the immune process, and the immune algorithm is to solve the optimal solution of NBP.

According to the working principle of immune algorithm, we can get the steps of immune algorithm:

1. Identification of antigen: the immune system can get and determine the information of antigen invasion
2. Producing the initial parent population: memory cells recognize and bind to antigens, and some of the best antibodies in the initial paternal population (the optimal solution of NBP) are selected from the database
3. Computational affinity: the matching degree between antibody and antigen was analyzed
4. Memory cell differentiation: the antibody that is most compatible with the antigen produced by (3) is presented to the memory cells, and those antibodies that are less compatible with the antigen will be replaced by the newly produced antibodies that match the antigen
5. Antibody promotion and inhibition: the immune system promotes antibodies that are highly compatible with the antigen and inhibits high-density antibodies similar to the antibody
6. Antibody renewal: for new antigens not touched by the immune system, the cleared antibodies by (5) will be replaced by lymphocytes, and various types of antibodies can be obtained by crossover mutation operator

The immune algorithm has the following characteristics:

1. Solving the diversity of candidates: for different candidate solutions, similar to the least square algorithm, the immune algorithm can obtain a global optimal solution for the problem to be optimized
2. Learning and memory: by learning and memory, an optimal global solution of NBP can be obtained quickly, that is, the immune system combines the antibodies with the invading antigens in a more rapid way and clears them away
3. Efficient parallel search: immune algorithm and genetic algorithm (GA) are both optimization model algorithms simulating biological physiological mechanism, but their underlying mechanisms are different. The difference between them can be summarized as follows [25, 26]:
4. From a biological point of view, GA is a competition between the evolution of individuals in a population and the heredity of their parents' genes. Immune algorithm is a kind of ability formed by an individual to adapt to the environment, the body to inhibit the invasion of external non-sels or remove their own pathological cells [27]
5. In the immune algorithm, antibodies and antigens, antibodies and different antibodies can interact with each other, forming a dynamic network system; GA does not consider the interaction between individuals
6. In immune algorithms, the body's genes can be optimized by themselves in some way; in GA, the changes in genes are determined by the environment
7. Genes in immune algorithms are carried out within the same organism, and the diversity is produced by the combination of genomes. GA often uses crossover operator, and the individual gene is the result of the crossover of the previous generation [28]

#### 3.3.2. Support Vector Machine

Support vector machine (SVM) was first proposed by V. Vapnik of AT&T Bell Laboratory. It is a machine learning method based on VC dimension theory of statistical learning theory and structural risk minimization principle. It has succinct mathematical form, intuitive geometric interpretation, and good generalization ability. It is a powerful tool to solve classification, regression, probability density estimation, and other issues [29]. It can automatically find the support vectors which have better distinguishing ability to classify, and the classifier constructed from this can maximize the distance between classes, so it has higher classification accuracy. The core content of support vector machine is mainly put forward in the 1990s. At present, the international discussion and further research on this theory are gradually widespread [30].

SVM is a new small sample learning method with solid theoretical foundation. It basically does not involve probability measure and law of large numbers, so it is different from the existing statistical methods. Essentially, it avoids the traditional process from induction to deduction, realizes efficient “transductive reasoning” from training samples to forecast samples, and greatly simplifies the usual classification and regression problems.

The final decision function of SVM is determined only by a few support vectors, and the complexity of calculation depends on the number of support vectors, not the dimension of sample space, which in a sense avoids the “dimension disaster.” A small number of support vectors determine the final result and help to grasp the key samples and “eliminate” a large number of redundant samples. Moreover, this method is not only simple but also has a good “robustness.” This “robustness” is mainly reflected in the following: adding or deleting nonsupport vector samples has no effect on the model, and support vector sample set has a certain robustness [31].

The main principles of support vector machines can be roughly summed up as the following two points:

1. The corresponding relationship between the independent variables and the strain variables is mapped from the original low-dimensional vector space to the high-dimensional vector space, making it a linear separable state, so that the nonlinear eigenvectors can be linearly analyzed in the high-dimensional feature space by using the linear algorithm
2. Based on the structural risk minimization principle, find a hyperplane in the feature space by means of an optimal tool to divide the data and its components into two categories to obtain the optimal classification effect

Simply put, the problem for SVM is to find a hyperplane and effectively separate two different classes of data [32, 33].

### 3.4. Ultrasonic Liver Image Classification and Recognition Based on Optimized Immune Algorithm

In this paper, the most commonly used immune algorithm for learning and optimal computing is combined with SVM. The speed and accuracy of SVM classification are improved by the concepts of replication, mutation, and selection in the processing to preserve the optimal antibody. Finally, an immune algorithm combined with SVM is formed. The basic process of the operation of the immune algorithm is shown in Figure 2.

Firstly, after extracting and calculating the eigenvalues of the ultrasound liver images, the accuracy of SVM is calculated and the affinity between antibodies and antigens is evaluated. If the stopping condition is not satisfied, this paper uses the immune algorithm to filter the features and select the parameters of support vector machine classification and then passes them to support vector machine for analysis and recognition.

Because SVM itself is very sensitive to noise and poor eigenvalues of training samples and if the multiple eigenvalues used in this paper are not properly screened, the accuracy of SVM for liver classification may be reduced. Therefore, this paper combines the immune algorithm and support vector machine to form an optimized immune algorithm which can improve the shortcomings of support vector machine and improve the accuracy of classification. The principle of this algorithm can be summed up as follows: firstly, the features before classification are brushed and the parameters of support vector machine are selected by immune algorithm so that the parameters *C* and *r* of radial basis kernel (RBF) can be transformed into higher dimensional space. The algorithm steps can be summarized as follows:

**Step 1 (initial antibody production).**

The immune algorithm first produces an array of binary encoded initial antibodies, in which a parameter is selected for each *n*-bit. The total length of a group of antibodies is 32∗*n* bits because each group of initial antibodies needs to select two parameters and thirty feature screening results of the support vector machine.

All the values in the binary initial antibody are selected by random number. After each parameter is generated, the original binary parameter is converted to decimal by the following formula:

(6) $$\begin{array}{c} x_{i}=d_{i}+\frac{u_{i}-d_{i}}{2^{l_{i}}-1}\left(\overset{l_{i}}{\underset{j=1}{\sum }}a_{j}2^{j-1}\right), \end{array}$$

where *x*_*i*_ is the value of every binary parameter converted to decimal, *u*_*i*_ and *d*_*i*_ are the upper and lower limits of the parameter, respectively, *l*_*i*_ is the length of each binary parameter, and *a*_*j*_ represents the value of the original binary parameter.

When all the parameters are decimal and then put into the support vector machine for calculation, the feature selection part will be randomly selected according to the given selection ratio. Finally, the recognition accuracy of the liver is regarded as the affinity between the antibody and antigen.

**Step 2 (replication and variation).**

After the affinity values of the initial antibodies and antigens in the first stage are calculated, the affinity values of these groups are first compared. The greater the affinity (that is, the higher the accuracy), the more likely this group of antibodies will have to replicate and mutate to find the optimal solution. Therefore, the size of antibody replicas with optimal affinity will be higher than that of generic antibodies. All the initial antibodies were duplicated and mutated by binary coding. The mutation rate was related to the coding length of each parameter in the binary initial antibody. The longer the given coding length was, the smaller the mutation probability was. The replicated and mutated antibodies are then converted to decimal in the same way and put into SVM.

**Step 3 (select the antibody with the best affinity).**

The replicated and mutated antibodies are then individually compared with their initial antibodies and retain the most affinity antibodies for the next cycle. The cycle of the entire optimized immune algorithm will last until the affinity reaches our desired goal or the number of cycles set.

## 4. Experiments

In the experimental simulation work, the computer hardware configuration is as follows:

1. Processor: Intel i5 2.50 GHz
2. Memory: 4 GB
3. Operating system: Windows 7 64 Ultimate
4. The simulation software is Matlab 2016b

## 5. Discussion

When extracting features from ultrasonic liver images, the image should be preprocessed in order to extract effective features and prevent the occurrence of false recognition caused by noise and other factors.  Figure 3(a) gives the grayscale image scanned by B-mode ultrasound, and the noise can be clearly seen from Figure 3(a) because of the equipment or other uncontrollable factors. In order to extract the image features better, this paper filters the image of Figure 3(a) and gets the image of Figure 3(b). Comparing the two images, it can be found that the features of Figure 3(b) are more obvious, and noise and other interference are effectively removed.

After filtering, the image is enhanced. The results are shown in Figure 4, in which Figure 4(a) is the result of filtering and Figure 4(b) is the result of image enhancement. From Figure 4, it can be seen that the gray level of the filtered image is relatively concentrated, and after image enhancement, the brightness of the image pixels is high or low, which makes the features of the ultrasound liver image more easily distinguishable.

Then, the image is binarized. The result is shown in Figure 5.  Figure 5(a) is the image before binarization, and Figure 5(b) is the image after binarization. As can be seen from Figure 5, after binarization of the image, the data volume of the algorithm is less, the image sensitive area can be highlighted, and the gray level of the whole image is reduced to the binary dimension, which greatly simplifies the subsequent feature extraction algorithm.

In this paper, a total of 300 samples of liver ultrasound images including 100 normal livers, 100 cirrhosis, and 100 hepatocellular carcinomas were randomly divided into five groups. One of the samples was selected by turns for testing, and the other four groups were used as training samples of support vector machine. The parameters of the immune algorithm optimized in this paper are as follows: the initial number of antibodies is 5 groups, the replication rate of general antibodies in each cycle is 10 times, the replication rate of antibodies with optimal affinity is 30 times, and the cycle algebra is 500 times.

In Figure 6, a graph of the affinity of the optimized immune algorithm with algebra is given. From the graph, it can be seen that the affinity value decreases rapidly in the first 50 cycles, which means that the algorithm is searching globally fast to get close to the optimal solution. In 50 to 250 cycles, the affinity value decreases slowly, which means that the algorithm searches locally to find the optimal solution near the optimal solution; after 250 cycles, the affinity value does not change, which indicates that the algorithm has found the optimal solution.

In order to better illustrate the advantages of the algorithm, this paper will use immune algorithm, support vector machine, and the immune algorithm optimized in this paper to identify and analyze the samples; data comparison is shown in Table 1; according to the data in Table 1, the accuracy of the three algorithms compared with the broken line graph is shown in Figure 7.

As can be seen from Table 1, (1) with the increase of the number of features, the recognition accuracy of the three algorithms is improved; (2) the number of execution times of immune algorithm is less than that of support vector machine, but its accuracy rate is much lower than that of support vector machine; (3) compared with the immune algorithm, the optimized immune algorithm improves the execution times and the accuracy rate; (4) compared with the support vector machine, the optimized immune algorithm improves the execution times and the accuracy rate. Phenomena (2)–(4) illustrate that the search ability of the optimized immune algorithm is better than that of the immune algorithm and SVM. It shows that the immune algorithm can brush the features before classification and select the parameters of SVM, which can improve the shortcomings of SVM and improve the accuracy of classification.

In addition, the dimensionality of SVM is reduced by filtering the PCA feature number. Therefore, this paper compares the PCA dimensionality reduction method with the immune algorithm proposed in this paper. The comparison data is shown in Table 2, and the accuracy polyline graph is shown in Figure 8.

As can be seen from Table 2, the three algorithms have the highest resolution accuracy for normal liver images, followed by cirrhosis and liver cancer, and the optimized immune algorithm has a higher accuracy than SVM and PCA.

## 6. Conclusions

At present, ultrasound is more and more widely used, such as B-ultrasound in medicine. However, the performance of ultrasonic image recognition still needs to be improved. Therefore, this paper proposes a method of ultrasonic image recognition based on immune algorithm, which is applied to medical ultrasonic liver image recognition. Aiming at the deficiency of classification and recognition of immune algorithm and support vector machine, an optimized immune algorithm is formed to classify and recognize the normal liver, liver cirrhosis, and liver cancer ultrasonic images. The simulation results show that the optimized immune algorithm can effectively improve the iteration times and accuracy of the immune algorithm and support vector machine, and the recognition accuracy is higher than that of the dimension reduction method of support vector machine by principal component analysis. Similarly, the simulation results show that the optimized immune algorithm performs better in the classification and recognition of normal liver, liver cirrhosis, and liver cancer ultrasound images. In conclusion, the optimized immune algorithm designed in this paper has great potential in the application of medical ultrasound liver image recognition. Because the immune system of an organism is extremely complex and precise, the theory of artificial immune system can be improved and simulated based on various theories of biological immune system. The algorithm used in this paper is based on the replication selection theory of immune system. In addition, there are many methods developed from other concepts of biological immune system, such as negative selection algorithm and artificial immune network, as well as applications combined with other famous algorithms. Therefore, in the follow-up research, we can try to use different artificial immune system theories combined with support vector machine, in order to better improve the operation efficiency of support vector machine and the accuracy of tumor recognition.

## Figures and Tables

**Figure 1:** Working principle of immune algorithm.

**Figure 2:** Flowchart of optimized immune algorithm.

**Figure 3:** Ultrasound liver image preprocessing.

**Figure 4:** Image enhancement processing.

**Figure 5:** Image binarization processing.

**Figure 6:** Change of affinity value with cycle number.

**Figure 7:** A broken line graph for comparing the accuracy of three algorithms.

**Figure 8:** Comparison of three algorithms for three liver discrimination accuracy rates.

**Table 1:** Comparison of three algorithms for recognition data.

Characteristic number	Immune algorithm		Support vector machine		Optimized immune algorithm	
	Number of execution	Accuracy	Number of execution	Accuracy	Number of execution	Accuracy
5	405	87.1%	1990	91.2%	250	94.13%
6	424	88.5%	3312	91.9%	277	94.63%
7	456	89.9%	7154	92.5%	312	96.12%

**Table 2:** Analysis of three kinds of liver data by three algorithms.

Ultrasound liver image	Accuracy		
	PCA dimension reduction method	Optimized immune algorithm	Support vector machine
Normal	97.9%	100%	98.21%
Cirrhosis	92.11%	94.13%	91.2%
Liver cancer	88.45%	93.34%	89.24%

## Data Availability

Data can be available on request.
